The article "Study of the Antimicrobial Activity of the Chinese Dong Ethnic Minority Medicine, Madeng'ai" was published in 2022. Journal: Evid Based Complement Alternat Med.

# Study of the Antimicrobial Activity of the Chinese Dong Ethnic Minority Medicine, Madeng'ai

**DOI:** 10.1155/2022/3678240

**Published:** 2022-08-01

**Authors:** Zhenrong Tang, Yannan Zhao, Zaiqi Zhang, Huan Yue, Dan Wang, Shengchun Liu, Hua Tang

**Affiliations:** ^1^Key Laboratory of Molecular Biology for Infectious Diseases (Ministry of Education), Institute for Viral Hepatitis, Department of Infectious Diseases, Chongqing 400016, China; ^2^Department of Endocrine and Breast Surgery, The First Affiliated Hospital of Chongqing Medical University, Chongqing 400016, China; ^3^Hunan Provincial Key Laboratory of Dong Medicine, Hunan University of Medicine, Hunan 418000, China

## Abstract

The overuse of antibiotics has contributed to the emergence of multidrug-resistant bacteria, which poses a challenging task for clinical therapy. Thus, new agents with antibiotic efficacy against multidrug-resistant infections are needed. The traditional Dong ethnic minority medicines have emerged as a new source for prodrug selection. Among them, Madeng'ai (*Potentillafreyniana*Bornm) is widely used by the folk for anti-infection and wound healing, although the mechanisms remain unclear. In this study, the antimicrobial activities of Dong medicine Madeng'ai were evaluated both *in vitro* and i*n vivo*. *S. aureus*, *E. coli*, *E. faecalis*, *P. aeruginosa*, *K. pneumoniae*, and *A. baumannii* were cultured in LB media, different concentrations of Madeng'ai powder solution were added to the LB agar plates to evaluate minimal inhibitory concentration. An animal study was performed on a mouse excisional wound model combined with bacterial solution injection in the wound area. After Madeng'ai or PBS treatment, hematoxylin and eosin analysis were used for pathological analysis of skin tissues from the infected area. Madeng'ai powder solution over 2 mg/mL concentration completely inhibited *E. coli* growth. At 4.0 mg/mL, Madeng'ai significantly inhibited the growth of *E. faecalis*, *Pseudomonas aeruginosa* (PAE), *Klebsiella pneumoniae*, and *Acinetobacter baumannii*. The mouse model revealed that Madeng'ai could suppress the growth of MRSA and PAE and accelerate healing of cutaneous wounds. Madeng'ai, a newly discovered Dong ethnic minority medicine possesses considerable antimicrobial activity against both human normal pathogenic bacteria and multiresistance bacteria such as *Pseudomonas aeruginosa, S. aureus,* and *Acinetobacter baumannii*. Therefore, Madeng'ai has great potential for further study and clinical application.

## 1. Introduction

Although a wide range of antibiotics have been developed, their overuse and misuse has led to the emergence of antimicrobial resistance (AMR), which is a threat to international public health [1, 2]. It is estimated that in Norway, Iceland, and the European Union, 25,000 AMR-associated deaths have occured annually since 2009, while in the USA, this number is estimated to be 99,000 [3, 4]. The threat of AMR in the USA is well documented in the CDC's report titled “Antibiotics Resistance Threats in the United States, 2013.” The UK's National Risk Assessment (NRA) reported that the number of AMR infections would continue to increase significantly. In China, the National Health and Family Planning Commission reported the “National Action Plan for Containing Antibacterial Resistance (2016–2020)” in 2016 [5].

The article "Study of the Antimicrobial Activity of the Chinese Dong Ethnic Minority Medicine, Madeng'ai" was published in 2022. Journal: Evid Based Complement Alternat Med.

AMR increases the risk of uncontrolled infection, sepsis, septic shock, microbial toxic syndrome, and even mortality. It is estimated that globally, there were 48.9 million cases of sepsis and 11 million sepsis deaths in 2017 [6]. In Japan, a prospective nationwide cohort study of sepsis carried out from 2016-2017 found that *E. coli* was the most common cause of sepsis, *S. aureus* was the most common Gram-positive bacteria, methicillin-resistant *S. aureus* (MRSA) was the most fatal bacteria, and that Gram-positive bacteria were slightly more common in sepsis than Gram-negative bacteria [7]. Goldstein et al. reported that the rates of sepsis-associated hospitalization and mortality have increased markedly in the last 2 decades. *E. coli* is the main cause of septicemia-associated hospitalization in patients aged >50 years and the main cause of mortality in adults (18–84 years old) [8]. A Chinese study by Chen et al. found that Gram-positive bacteria are as prevalent as Gram-negative bacteria in adults with sepsis and that in neonates, sepsis from Gram-positive bacteria was more common than sepsis from Gram-negative bacteria [9]. Thus, it is crucial to monitor the development of antimicrobial resistance. Novel antimicrobial agents with efficacy against AMR strains are urgently needed [2, 10].

Natural products have served as a major source of antibacterial agents. For instance, honey has been used for millennia as a topical treatment for wounds and burns. Manuka honey is reported to inhibit a wide range of microorganisms [10]. *Artemisia argyi* (Chinese mugwort) has been used as a traditional Chinese herbal medicine for millennia. Xiao et al. reported that *Artemisia argyiLevl. et Vant* essential oil extracted through simultaneous distillation has high antimicrobial activity against *L. monocytogenes, E. coli,* P. Vulgaris*, S. enteritidis, and A. Niger* [11]. It is reported that leaf extracts from *Potentilla fruticosa, Potentilla glabra, and Potentilla parvifolia*, traditional Chinese herbs of the *Rosaceae* family, possess significant microbial inhibition effects [12]. *Potentilla fruticosa* was the most potent inhibitor of Gram-positive bacteria and *P. aeruginosa*, while *Potentilla parvifolia* exhibited broad-spectrum antifungal and antibacterial effects [12]. These reports indicate that some herbs and natural products have great potential for antimicrobial use. *Potenllia freyniana Bornm*, a member of the genus *Potenllia* and family *Rosaceae*, is widely distributed in southern China provinces, including in Hunan, Guizhou, and Guangxi. Madeng'ai (Figure 1) is a variant of *Potenllia freyniana Bornm*, and has long been medicinally used by the Chinese Dong ethnic minority for the treatment of infection, wound healing, and empyrosis. This phenomenon inspires us that Madeng'ai may have beneficial effects on human pathogenic bacteria infection, although no relevant study has been published. Due to the widespread drug resistance, new chemicals or herbal medicines are urgently needed for the treatment of antimicrobial resistant (AMR) infections. For instance, methylene blue has now been proven to be highly effective in inhibiting the growth of *Mycobacterium tuberculosis* [13]. In this study, using *in vitro* and *in vivo* studies, we showed that Madeng'aihas antimicrobial activity on human normal pathogenic and multiresistant bacteria, and this Dong medicine has great potential for further study and application.

The article "Study of the Antimicrobial Activity of the Chinese Dong Ethnic Minority Medicine, Madeng'ai" was published in 2022. Journal: Evid Based Complement Alternat Med.

## 2. Materials and Methods

### 2.1. Plant Materials

Madeng'ai samples were collected from a grassland 800 meters above sea level, in Tongdao County, Huaihua City, Hunan Province, and identified by the Hunan Provincial Key Laboratory of Dong Medicine, Hunan University of Medicine according to its growing area, botany morphology of leaf, root, stem, and flower color, and other comprehensive factors. The plant materials were powdered and stored at 4°C until use.

### 2.2. Microorganisms

*Staphylococcus aureus* (*S. aureus*, ATCC25923), *Escherichia coli* (*E. coli,* ATCC259220), *Enterococcus faecalis* (*E. faecalis,* ATCC29212), *Pseudomonas aeruginosa* (*P. aeruginosa,* ATCC2785), *Klebsiella pneumonia* (*K. pneumoniae*) and *Acinetobacter baumannii* (*A. baumannii*) were obtained from the First Affiliated Hospital of Chongqing Medical University, China. The latter two bacteria were isolated from patients' sputum and belong to nonmultiple drug-resistant bacteria based on drug susceptibility tests (using the minimum inhibitory concentration method).

### 2.3. Minimum Inhibitory Concentration (MIC) Evaluation

MIC refers to the lowest concentration of extracts capable of inhibiting visible bacterial growth. According our preliminary study, Madeng'ai powder (0, 100, 200, 300, 400, and 500 mg) was added into flasks containing 100 mL of LB broth media and autoclaved to generate 0, 1, 2, 3, 4, and 5 mg/mL Madeng'ai extract suspensions. Next, 100 *μ*L aliquots of MRSA or E.coli cultures with a density of 5 × 105 CFU/mL (0.5 McFarland method) were added to the 100 μL LB broth containing different Madeng'ai extracts and cultured overnight, 37°C, with shaking at 220 rpm for 2-3 hours until an OD600 (Optical Density) of 0.5 was reached in low concentration of Madeng'ai extract groups. Finally, 100 *μ*L aliquots from the 6 cultures of MRSA or E.coli were spread on normal LB agar plates and cultured overnight. The inhibitory role of Madeng'ai extracts on bacteria was judged by the naked eye, ignoring single colony within the area of the inoculated spot.

The article "Study of the Antimicrobial Activity of the Chinese Dong Ethnic Minority Medicine, Madeng'ai" was published in 2022. Journal: Evid Based Complement Alternat Med.

### 2.4. Antibacterial Activity Evaluation in Animal Experiments

tMouse experiments adhered to the animal use guidelines of the National Institutes of Health and were approved by the Ethics Committee for Animal Experiments of Chongqing Medical University. All mice were housed in laminar flow cabinets under specific pathogen-free conditions at room temperature with a 12 h light/dark cycle and with *ad libitum* access to food and water. Twelve female BABL/c mice (5–6 weeks old) were randomly divided into the MRSA-medicine, MRSA-PBS, PAE-medicine, and PAE-PBS groups. Next, the backs of the mice were shaved and a 0.5 cm diameter wound was made using a sterile surgical scissor. Methicillin-resistant *Staphylococcus aureus* and *P. aeruginosa* were cultured in LB broth at 37°C with shaking at 220 rpm for 2–3 hours until an OD600 nm value of 0.5 was reached. The viable count of microorganisms was measured by the plate counting method and adjusted to a density equivalent to 10^6^ CFU/ml. A 100 *μ*L suspension of MRSA or PAE was then subcutaneously injected into the wound area within 30 min to avoid changes in inoculum density. For animal studies, powdered Madeng'ai (10 g) root was added to 50 mL of autoclaved Milli-Q water and autoclaved to generate a pasty suspension (concentration: 0.2 g/mL). After 48 h, the Madeng'ai extract was applied twice daily on the wound surfaces of the MRSA/PAE-medicine group using a cotton swab. PBS was similarly applied to the wounds of the MRSA/PAE-PBS group.

### 2.5. Wound Recovery and Changes in Mice Weight

The weight of the mice and the rate of recovery were monitored daily for 10 days after wound treatment with the Madeng'ai extracts and PBS control.

### 2.6. Rate of Bacteria Growth and Histological Analysis after Treatment

After wound treatment with Madeng'ai or PBS for 10 days, wound regions were disinfected with 75% ethanol. The wound surfaces were then cut down with sterile surgical scissors and swabbed on LB agar plates for bacteria culture. Wound surfaces were then sectioned at 4 *μ*m and stained with H&E for histological analysis.

The article "Study of the Antimicrobial Activity of the Chinese Dong Ethnic Minority Medicine, Madeng'ai" was published in 2022. Journal: Evid Based Complement Alternat Med.

### 2.7. Statistical Analysis

Data are presented as the mean ± standard deviation (mean ± SD), and analyzed by SPSS software for Windows (version 23.0). A comparison of means between groups were performed by the Student's *t*-test. Differences among the experimental groups were analyzed by one-way analyses of variance followed by LSD or Dunnett's T post hoc test. *p* < 0.05 was considered significant.

## 3. Results

### 3.1. Minimum Inhibitor Concentration (MIC)

The antimicrobial activities (MIC values) of Medeng'ai against common Gram-positive and Gram-negative bacteria are shown on Figure 2. For *S. aureus,* Madeng'ai exhibited macroscopic inhibitory activity at 2 mg/mL as almost no macroscopic *S. aureus* colonies were observed at this concentration. At 1 mg/mL, Madeng'ai suppressed the growth of *S. aureus* LB agar plates as fewer *S. aureus* colonies were observed relative to untreated cultures. Madeng'ai extracts also inhibited the growth of *E. coli* on LB agar plates with the strongest inhibition observed at 4 mg/mL with no observable macroscopic *E. coli* colonies. Although 1 mg/mL of the extract suppressed *E. coli*, 2 and 3 mg/mL almost completely inhibited *E. coli* growth on LB agar plates when compared to untreated controls.

To determine its antimicrobial spectrum, its inhibitory effect was examined against various bacteria on an LB agar plate (Figure 3). This analysis showed that 4.0 mg/mL Madeng'ai had macroscopic inhibitory activity against *E. faecalis* (Gram-positive) and *P. aeruginosa* (Gram-negative) as well as against *K. pneumoniae* and *A. baumannii* (both Gram-negative), isolated from patients' sputum.

### 3.2. *In vivo* Antimicrobial Activity

The wound healing rates in the MRSA-medicine and MRSA-PBS groups are shown in Figure 4. On Day 0 (before treatment), infected wound areas were obviously visible in both the MRSA-medicine group and the MRSA-PBS group. However, on Day 6 (after treatment), the wound areas in the MRSA-medicine group were markedly smaller when compared to Day 2. Moreover, wound margins were more distinct and regular on Day 6 when compared to Day 2 and wound secretions were reduced relative to Day 2. In contrast, on Day 6, mice in the MRSA-PBS group (MRSA untreated) had larger infected wound areas than on Day 2. Moreover, wound margins were less well-defined on Day 6 when compared to Day 2 and wound secretions were increased relative to Day 2. On Day 10, the wounds on MRSA-medicine mice were markedly healed and had no redness, swelling, or macroscopic wound area when compared to MRSA-PBS mice, whose wounds were still infected, open, red in color, and swollen.

The article "Study of the Antimicrobial Activity of the Chinese Dong Ethnic Minority Medicine, Madeng'ai" was published in 2022. Journal: Evid Based Complement Alternat Med.

The wound healing status of the PAE-medicine and PAE-PBS groups are shown on Figure 5(a). The results revealed that the infected wound recovered better in the PAE-medicine group when compared to the PAE-PBS group. On Day 0 (before treatment), infected wound areas were obviously visible in both the PAE-medicine group and PAE-PBS groups. However, on treatment Day 6, the infected wound area in the PAE-medicine group was smaller than on Day 2. Moreover, the infected wound margin was more defined and regular, and the wound secretions were reduced when compared to Day 2. On Day 10, the wounds on PAE-medicine mice had clearly healed and did not have redness, swelling, or macroscopic wound area when compared to PAE-PBS mice whose wounds were still infected, red, swollen, and open.

### 3.3. Bacterial Growth Condition and Histological Analysis after Treatment

The growth rates of infected bacteria from wound secretions after MRSA and PAE treatment surfaces (recovered or unrecovered) are shown in Figures 4(b) and 5(b), respectively. Very few bacterial colonies were observed upon culturing bacteria from MRSA-infected wounds treated with Madeng'ai extracts on LB agar plate. However, numerous MRSA colonies were observed upon culturing bacteria from the wounds of PBS-treated mice. Similar observations were made upon culturing bacteria from PAE-infected wounds when compared to bacteria cultured from the wounds of PBS-treated mice.

H&E analyses of wound surfaces (recovered or unrecovered) after treatment revealed vast numbers of inflammatory cells (bluish-violet cells marked with red circles) were observed on the upper pictures of both (Figures 4(c) and 5(c)), indicating that MRSA/PAE wound infection persisted after PBS treatment. However, the number of inflammatory cells was markedly reduced upon treatment of MRSA- and PAE-infected wounds with Maadeng'ai extract. Moreover, the epidermis was more intact in treated animals than in PBS controls, indicating that Madeng'ai promoted the healing of infected wounds (Figures 4(c) and 5(c)). No obvious changes in mouse body weight were noticed during the treatment period (Figures 4(d) and 5(d)).

## 4. Discussion

In this study, we show that on LB agar plates, 2 mg/mL of Madeng'ai markedly inhibits the growth of *S. aureus* and *E. coli*, respectively. Moreover, our data show that the extract has broad spectrum activity at a MIC of 4 mg/mL against Gram-positive and Gram-negative bacteria. Further analysis revealed that at 4 mg/mL, the extract could also inhibit the growth of other common infectious bacteria, including *E. faecalis*, PAE, *K. pneumoniae*, and *A. baumannii*. It should be noted that the 0, 1, 2, 3, 4, and 5 mg/mL of Madeng'ai extracts we used in this study is the concentration of crude herb powder rather than herb extracts or pure compounds. Since the Madeng'ai powder or boiled soup was traditionally used by the Dong and Miao ethnic minorities of China as analgesic and antibacterial agents, we believe the active ingredients could be extracted during the autoclaving process (20 mins). Although some active compounds may be inactive during this process, and the extract efficiency may not be high due to the short extraction time, the data reported in this work is promising. The antibacterial activities of water and alcohol extracts of Madeng'ai under various conditions and the active compounds responsible for the antibacterial activities should be investigated in further study. Crucially, mouse experiments revealed that the Madeng'ai extract has strong antimicrobial activity against methicillin-resistant *S. aureus* and PAE and promoted wound healing in mice compared to untreated controls. Moreover, bacterial culture results revealed that negligible levels of MRSA and PAE existed in the secretions of Madeng'ai treated mice. H&E analysis revealed that treatment with Madeng'ai reduced inflammatory infiltration and promoted skin regeneration in the wound area.

The article "Study of the Antimicrobial Activity of the Chinese Dong Ethnic Minority Medicine, Madeng'ai" was published in 2022. Journal: Evid Based Complement Alternat Med.

Large numbers of drugs with antimicrobial activity have been discovered and deployed clinically. Anne H. Norris and colleagues recommended that the choice of antimicrobial agents be based more on the outpatient parenteral antimicrobial therapy model than on the drug's pharmacokinetics [14]. Antibiotics like vancomycin, cefazolin, or aminoglycosides may be limited to patients who receive parenteral antimicrobials during dialysis sessions [15]. Li et al. showed that decisions on antimicrobial prophylaxis should be based on contamination in the surgical field. For instance, antibiotics should be used to prevent postoperative surgical site infection, which is mainly caused by *S. aureus*. Besides, before colon and rectal surgery, antibiotics were also applied to combat the infections may be caused by *E. coli* [16]. Empirical therapy for bacterial infections is widely accepted because it is effective. For instance, vancomycin and antistaphylococcal penicillin are used empirically to inhibit *S. aureus* bacteremia and vancomycin is the first choice treatment for MRSA [17, 18]. Fosfomycin-trometamol and nitrofurantoin have been recommended as first-line antibiotics for uncomplicated cystitis. Fluoroquinolones are first-line oral treatments for uncomplicated pyelonephritis as well as for *E. coli,* the leading cause of uncomplicated urinary tract infection [19–21].

The article "Study of the Antimicrobial Activity of the Chinese Dong Ethnic Minority Medicine, Madeng'ai" was published in 2022. Journal: Evid Based Complement Alternat Med.

However, the development of antibiotics has been accompanied by antimicrobial resistance, and mounting effort has gone into understanding the mechanisms of antimicrobial resistance. Antimicrobial resistance may happen when the target cell's wall is poorly permeable or permeability is specifically reduced for a given antibiotic [22]. Resistance may also result from loss of chemical affinity between an antimicrobial agent and its target, as happens in streptococci [23]. Additionally, antimicrobial activity may be suppressed by the bacterium, as happens in *β*-lactamase production [24]. Other mechanisms of antimicrobial resistance include the extrusion of antimicrobial agents from bacterial cells by efflux systems [25] and the production of extracellular polymer substances in biofilms that may impair the diffusion of antimicrobial agents through electrostatic and steric interactions [26]. Thus, novel, effective antimicrobials are urgently needed.

Although we have not determined the antimicrobial mechanism of Madeng'ai, numerous studies have indicated the antimicrobial role of *Potentilla* species attributed to their phenolic compounds [12, 27]. Thus, future studies should investigate the underlying mechanisms of the antimicrobial activity of Madeng'ai. Furthermore, because of their anti-inflammatory and vasoconstrictive effects, *Potentilla* species are used to treat topical inflammatory skin disorders [28–30] and diabetes mellitus [31, 32]. Therefore, the therapeutic potential of Madeng'ai against microbial infections and other diseases warrants further investigation.

## 5. Conclusion

Taken together, Dong ethnic minority medicine Madeng'ai possesses antimicrobial activity against both human normal pathogenic bacteria but also multiresistance bacteria such as *Pseudomonas aeruginosa*, *S. aureus*, and *Acinetobacter baumannii*. Therefore, Madeng'ai has great potential for further study and application.

## Figures and Tables

**Figure 1:** Morphology of Madeng'ai, a variant of *Potentilla freyniana Bornm* (lower panel) and *Potentilla freyniana Bornm* (upper panel).

**Figure 2:** (a) MIC results of Madeng'ai against *S. aureus* and *E. coli*. (b) The number of colonies on plates of different concentrations of Madeng'ai against *S. aureus* and *E. coli*. ^*∗∗∗*^*p* < 0.01 versus blank control group.

**Figure 3:** (a) The inhibitory effect of Madeng'ai against *E. faecalis*, *P. aeruginosa* (PAE), *K. pneumoniae,* and *A. baumannii*. (b)The number of colonies on plates of *E. faecalis*, *P. aeruginosa* (PAE), *K. pneumoniae,* and *A. baumannii* after 4 mg/ml Madeng'ai treatment. ^*∗∗∗*^*p* < 0.01 versus blank control group.

The article "Study of the Antimicrobial Activity of the Chinese Dong Ethnic Minority Medicine, Madeng'ai" was published in 2022. Journal: Evid Based Complement Alternat Med.

**Figure 4:** The effects of Madeng'ai on bacterial growth and histological and body change of methicillin-resistant *S. aureus*-infected mice. (a) Recovery of methicillin-resistant *S. aureus*-infected wounds on BALB/c mice after Madeng'ai or PBS treatment. (b) LB agar of methicillin-resistant *S. aureus* growth from infected wound secretions after treatment with Madeng'ai or PBS. (c) H&E analysis of skin tissues from wounds infected with methicillin-resistant *S. aureus* after treatment with Madeng'ai or PBS. (d) Changes in mouse body weight during treatment.

**Figure 5:** The effects of Madeng'ai on bacterial growth and histological and body change of PAE-infected mice. (a) Recovery of PAE-infected wounds after treatment with Madeng'ai or PBS (control). (b) The growth of PAE from wound secretions of infected mouse. (c) H&E analysis of skin tissues from wounds infected with PAE after treatment with Madeng'ai or PBS (control). (d) Changes in mouse body weight during treatment.

## Data Availability

All data used to support the findings of this study are included within the article.

## Abbreviations

AMR: Antimicrobial resistance
MIC: Minimum inhibitory concentration
MRSA: Methicillin-resistant *Staphylococcus* aureus
*E. coli*: Escherichia coli
PAE: Pseudomonas aeruginosa
*K. pneumoniae*: Klebsiella pneumoniae
*A. baumannii*: Acinetobacter baumannii
*E. faecalis*: Enterococcus faecalis
*S. aureus*: Staphylococcus aureus.
